# Computational Models-Based Detection of Peripheral Malarial Parasites in Blood Smears

**DOI:** 10.1155/2022/9171343

**Published:** 2022-06-08

**Authors:** Amal H. Alharbi, C. V. Aravinda, Jyothi Shetty, Mohamed Yaseen Jabarulla, K. B. Sudeepa, Sitesh Kumar Singh

**Affiliations:** ^1^Department of Computer Sciences, College of Computer and Information Sciences, Princess Nourah bint Abdulrahman University, P.O. Box 84428, Riyadh 11671, Saudi Arabia; ^2^NITTE Deemed to Be University, Mangalore, India; ^3^School of Electrical Engineering and Computer Science, Gwangju Institute of Science and Technology (GIST), Gwangju, Republic of Korea; ^4^Department of Civil Engineering, Wollega University, Nekemte, Oromia, Ethiopia

## Abstract

The most common human parasite as per the medical experts is the malarial disease, which is caused by a protozoan parasite, and Plasmodium falciparum, a common parasite in humans. A microscopist with expertise in malaria diagnosis must conduct this complex procedure to identify the stages of infection. This epidemic is an ongoing disease in some parts of the world, which is commonly found. A Kaggle repository was used to upload the data collected from the NIH portal. The dataset contains 27558 samples, of which 13779 samples carry parasites and 13779 samples do not. This paper focuses on two of the most common deep transfer learning methods. Unlike other feature extractors, VGG-19's fine-tuning and pretraining made it an ideal feature extractor. Several image classification models, including VGG-19, have been pretrained on larger datasets. Additionally, deep learning strategies based on pretrained models are proposed for detecting malarial parasite cases in the early stages, in addition to an accuracy rating of 98.34^*∗*^ 0.51%.

## 1. Introduction

The leading cause of infection in all parts of the world is malaria, a deadly disease. The rapid consumption and high mortality rate of this epidemic condition have been documented throughout history. The global death toll from malaria was estimated at 4,29,000. In 2015, there were an estimated 3,03,000 children under the age of five years, and prenatal women are the most at risk of death [1]. By detecting this disease at an early stage, the death rate can be reduced and prevented. Researchers face a challenge in providing the most accurate parasite detection in the shortest amount of time, cost, and effort. During the last few decades, this visual inspection has played a vital role in being a tool in the health check field for decision making. A thick blood smear can identify malaria parasites in blood samples [2]. This shows that it is close to eleven times more sensitive than a thin blood smear for the rapid detection of parasites. It is often used to test the development stages to create blood smears placed on a microscope glass slide. To confirm malaria infection, a pathologist uses a light microscope to identify changes in the size, shape, and perception of various RBCs. The pathologist's understanding of the disease depends on the accuracy of a plasmodium microscopic report. This technique is arduous and inefficient due to uncertainty, which can cause erroneous and contradictory diagnoses, as well as inappropriate medication and, in rare situations, the death of the patient and specimens of infected and noninfected microbes.

A mechanism for detecting malaria infection has been proposed using supervised learning. The methods for detecting malaria parasites were demonstrated by using in vitro culture image samples [3]. The samples developed in a laboratory do not contain substances other than WBCs, platelets, or parasites. When considering the severity of malaria depending on the number of deaths caused by the disease, it is reasonable to accept possible minor errors caused by an automated method during execution [4, 5]. Since the advent of deep learning techniques, feature extraction has been made far more efficient than traditional methods. Because deep learning methods still require trained experts and advanced techniques for calculating disease prediction, most of these methods still require efficient feature extraction optimization. There are many layers and levels of nonlinear mapping in CAD schemes based on ANN architecture. As a result of the layer-wise network of hidden layers, gradient-based optimization produces poor results [6, 7]. Microscopic diagnosis requires extensive training, experience, and skills. In rural areas where malaria is prevalent, manual microscopy has not proven to be an effective screening tool when performed by nonexperts [8–10]. This model was intended to enhance the model's performance by modifying the network architecture and hyper-tuning the features to achieve a better-performing model. To determine the key features in the future, this paper focuses on the network architecture. The basic VGG-19 model obtains 85% accuracy, but after fine-tuning the model and applying the data augmentation technique to the training dataset, it can attain 97.14%.

The following is the sequence under which this manuscript is structured.  Section 2 represents the related work and data acquisition.  Section 3 illustrates the proposed deep transfer learning methodology.  Section 4 discusses the findings.  Section 5 concludes the paper.

## 2. Related Work

There are several methods of identifying parasite RBCs. Purwar et al. preprocessed by utilizing local histograms [11]. The Hough transform and morphological operations are used for segmentation and classification of diseased and clean cells. Di Ruberto et al. employed a statistical k-means clustering algorithm [12]. Using thresholding, Ritter and Cooper [13] have segmented cells, separated overlaps, and modified division lines according to Dijkstra's algorithm. Diaz et al. [14] applied efficiency to develop templates from parasite-stained images, which would then be used to classify each cell's infection life stages. RBCs can be segmented from the background in blood images using a variety of techniques. Díaz et al. [15] determined whether the RBCs were infected by the parasite from the host or not by separating them. Savkare et al. [16] and Ross et al. [17] analyzed grayscale images using k-means and k-medians to define the overall clusters into two parts. The significance of supervised learning is to identify classes of sample data. These disease stages were identified with a blend of ML algorithms. Krizhevsky et al. [18] built a well-known CNN architecture, that is, the ALEX net, to compete with ImageNet and bagged awards. Quinn et al. [19] compared the CNN with a classifier using trees, and the accuracy rate was determined by analyzing the middle of the operating region. To identify blood cells on blood smear images, Chowdhury et al. [20] adopted a CNN approach to detect infections that were affected by the blood smears. Raviraja et al. [6] analyzed pretrained CNN models for malaria detection in blood cell images, namely, DenseNet121, VGG-16, Alexnet, ResNet50, FastAI, and ResNet101, Meng et al. [21]. With a high precision of 97.5%, ResNet50 excelled over the other CNN models [22]. To conclude, many deep learning algorithms for detecting malaria using cell images have been presented by Yue [23]. Many of them used large pre-trained CNN models to enhance the accuracy of classification, whereas others used customized CNNs to minimize the computational time [24].

The implications of substantial quantities of improperly classified data in medical image classification are catastrophic, and the objective of proposing a medical diagnosis tool is wrecked. In addition to efficiency, additional parameters such as F1 score [25, 26], area under the curve (AUC) [27, 28], sensitivity [29, 30], and specificity [31–33] are vital in analyzing various approaches. A random sample of cell images infected/not infected with malaria is shown in Figure 1.

### 2.1. Data Acquisition

The data was obtained from the National Institutes of Health portal and uploaded to a Kaggle repository. There are 27558 cell images in the dataset, out of which 13779 are malaria-infected cell images and another 13779 are malaria-free cell images. The random samples were collected and separated into three sets: training, testing, and validation. Next, 8000 images were deployed for training and 3000 images for validation for each class. These 11000 images have been used to train models. Subsequently, these were used along with the remaining 2779 images for each class as test data to evaluate the proposed models to perform on images that have never been seen before, because the original dataset included images with different dimensions, and it was scaled to equal dimensions before splitting the data. Most of the images were scaled to 128 × 128 pixels with three channels of RGB. Having all images equal will allow the neural networks to learn more quickly and with minimal mistakes in the future. The outcomes obtained excelled all existing methods, so data augmentation was used to improve the results. A few of the images in the class folders at the beginning are significantly different than the ones at the end. As a result, this was used to sample the data at random, as this will allow the proposed models to learn more diversified features from both classes, which will reduce overfitting and make our model more extensible to data.

## 3. Proposed Model

Morphological image processing is used to eliminate noise and recreate object features (see Figure 2). To achieve deep feature extraction and transfer learning, the convolutional layers are frozen. To classify RBCs, a fine-tuned pretrained CNN model with image augmentation is proposed (see Figure 3).

### 3.1. Transfer Learning

The paths, according to K. Fukushima, are the beginning of a deep convolutional neural network architecture. The idea has been around for a while, but due to the lack of efficient high computational power, it has yet to gain momentum. In recent times, graphics processing units have advanced significantly toward high-performance computing technologies. Computational intelligence techniques have gained prominence as a result of their high possibility. CNN is the most popular type of this approach, which is composed of the layers described below.

Three main CNN layers were used in this algorithm, namely, “convolution,” “pooling,” and “fully connected layers.” Figure 3 exhibits a schematic representation of a model with one conventional layer and one maximum layer. In the feature map, activation functions are used to increase the nonlinearity of the network ReLU. A neuron with the sigmoid activation function appears in the output layer of the model. When all negative values in the activation map are replaced with zero, ReLU activation completely cancels out all negative values. A binary classification model is built using sigmoid activation with a loss of function of binary cross-entropy. It has a learning rate of 0.01. In this case, the function gives a value between 0 and 1. Following the compilation of the dataset, the model will be trained based on the inputs received from the training samples, which will map the inputs to the outputs. It is a matter of choosing a set of weights that is best suited for resolving these problems.

### 3.2. Predictable Method

The initial model is trained by this network model using traditional methods of training for a given number of epochs. Model accuracies of 99.80% during training and 95.60% during validation were unchanged. Figures 4 and 5 show the exactness and failure graphs of the model. AUC score, specificity, sensitivity, and test accuracy were used to evaluate the performance.  Table 1 depicts an implementation of the test set, whereas Table 2 exhibits CNN model architecture. The input layer *a* = *i*1 and output layer io1 = 3 and *p*1 = 0, input layer c2d, output layer co1 = 32 and *p*1 = 896, max input layer mp2d and output layer mo2 = 32, and *p*1 = 0. The input layer c2d1, output layer c2do1 = 64 and *p*2 = 18496, and the input layer mp2d1 and output layer mpo1 = 64 and *p*2 = 0. The input layer c2d2, output layer c2o2 = 128, and *p*3 = 73856. The input layer = *m*2d2, output layer = *m*2do2 = 128, and *p*4 = 0. The input layer flattened layer = Fl, output layer flo = 28800, and *p*4 = 0. Input the dense layer dl, output layer det5 = 512, and *p*5 = 14746112. The input layer dropout = dot, output layer dot5 = 512, and *p*5 = 0. The input layer dns_1 and output layer dnst5 = 512 and *p*6 = 262656.

### 3.3. Pretrained CNN Model

Figures 6 and 7, respectively, demonstrate the accuracy model and performance for the VGG-19 pretrained model and weights as displayed in Table 3. The convolutional layers are divided into sixteen layers, and there are 3 ∗ 3 convolutional filters. The input layer b1-c1, output layer *t*1 = 64 and parameter *p*1 = 1792, the input layer b1-c2, output layer *t*1 = 64 and parameter *p*1 = 3698, and b1_pool and output *t*1 = 64 and parameter *p*1 = 0. The input layer b2-c1, the output layer *t*2 = 128, and the parameter *p*2 = 73856. The input layer b2-c2, the output layer *t*1 = 128, and parameters *p*1 = 147584 and b2_pool and output *t*2 = 1284 and parameter *p*2 = 0. The input layer b3-c1, output layer *t*3 = 256, and parameters *p*3 = 295168, b3_c2 output layer *t*3 = 256, and *p*3 = 590080, b3-c3 and b3-c4 output layer *t*3 = 256, and output layer *p*4 = 590080. The b3-pool and output *t*3 = 256 and *p*3 = 0. The input layer b4-c1, the output layer *t*4 = 512, and *p*4 = 1180160. The input layer b4-c2, b4-c3, b4-*c*4 = 512 and *p*4 = 2359808. The input layer b4-pool and *t*4 = 512 and the output layer *p*4 = 0. The input layer b5-c1, b5-c2, b5-c3, b5-c4, and *t*5 = 512, and the output layer *p*5 = 2359808. The input layer fla-1 and the output layer *t*5 = 4608 and *p*5 = 0. The input layer dse3 and output layer dset = 512 and *p*5 = 2359808. The input layer dtt2 and the output layer dtt5 = 512 and *p*5 = 0. The input layer dse4 and output layer dset5 = 512 and *p*5 = 262656. In addition to that, there are max pooling filters for downscaling and two fully connected hidden layers with 4096 units each. The remaining dense layer consists of one thousand units, each representing one of the image categories in ImageNet. The dense layer is fully connected, so the last three layers are skipped, and the five layers are concentrated to use the vgg19 model for feature extraction. This model was built from scratch using the original datasets that include all 19 trainable layers. The ReLU served as the activation function for the network. The Adam optimization was used to create the loss function. The model was built using transfer learning and using pre-trained frozen layers. Later, this model was used to generate the output of the images. This was implemented using the sigmoid activation function as a simple feature extractor by freezing all five convolutional blocks to prevent the weights from moving across epochs. This third model is fine-tuned and is built by freezing the first three blocks from the image net and then training blocks four and five from the malarial datasets. To fine-tune the VGG-model, blocks 4 and 5 were changed so that their weights are updated each time the model is evaluated. These preprocessing strategies were applied to this model, which includes normalization, data augmentation, and standardization. A sigmoid activation function with two methods was applied to solve the classification problem to gain an output of 1 for infected and 0 for healthy.

### 3.4. Image Augmentation with a Fine-Tuned Pretrained Model

In Figure 8, the existing images from the training samples were reworked and transformed to create a new, modified version of the originals because of rotation, shearing, translation, zooming, and so on. Figures 6 and 7 illustrate how the random transformation, model accuracy, and loss of the model are what are required to obtain the same images every time. The augmentation of the model accuracy is shown in Figures 9 and 10.

The confusion matrix (FN) is used to evaluate the number of positive and negative predictions as shown in Figure 11. The confusion matrix is used to determine whether a prediction is a truly positive or true negative.

## 4. Discussion

Individual red blood cell smear images are investigated to evaluate if they are infected or healthy. The study comprises a range of pretrained convolutional neural networks with transfer learning that are fine-tuned and registered on the malaria dataset. On VGG-19 and Transfer Learning, research shows that different preprocessing approaches like normalization and scaling do not affect model performance, however, the data augmentation technique has shown encouraging outcomes. The basic VGG-19 model obtains 85% accuracy, but after fine-tuning the model and applying the data augmentation technique to the training dataset, it can attain 97.14%, as shown in Table 4. Transfer learning is a wonderful strategy that can be used to create promising results, according to the research and the performance analyses depicted in Table 5.

## 5. Conclusion

The deep learning neural network model was applied to improve the model's performance. It was shown that standardization and normalization had less impact on classification. The use of data augmentation improved the model performance and yielded positive results. Models of VGG-19 and ImageNet were derived from the initial concept using the combination of transfer learning and parameter tuning. To determine the key features, this paper has focused on the network architecture. This was intended to enhance the model's performance by modifying the network architecture and hyper-tuning the features to achieve a better-performing model.

## Figures and Tables

**Figure 1:** A random sample of cell images infected/not infected with malaria [2].

**Figure 2:** Morphological filters applied to malaria cells.

**Figure 3:** Proposed CNN-model.

**Figure 4:** Model accuracy performance of CNN model.

**Figure 5:** Model loss performance of CNN model.

**Figure 6:** Accuracy performance of modified CNN model.

**Figure 7:** Loss performance of modified CNN model.

**Figure 8:** Sample augmented images.

**Figure 9:** Augmentation accuracy results.

**Figure 10:** Augmentation loss results.

**Figure 11:** Confusion matrix results.

**Table 1:** Performance test.

Metrics	Performance (%)
Testing-accuracy	95.56
F1 Score	96.45
A∪C score	95.45
Sensitivity	96.65
Specificity	95.25

**Table 2:** Convolution neural network model.

Layer	Output	Parameter
i_1	[(*N*, 125, 125, io1)]	*P*0
c2d	(*N*, 125, 125, co1)	*P*1
mp2d	(*N*, 62, 62, mpo2)	*p*01
c2d_1	(*N*, 62, 62, c2do1)	*P*2
mp2d _1	(*N*, 31, 31, mp2o1)	*p*02
c2d2	(*N*, 31, 31, c2o2)	*P*3
m2d_2	(*N*, 15, 15, m2do)	*p*03
Fl	(*N*, flo)	*P*4
Dl	(*N*, det5)	14746112
Dt	(*N*, dot5)	*p*05
dns_1	(*N*, dnst5)	262656
Dot	(*N*, dot5)	d05
dense_2	(*N*, 1)	513
Total	—	15,102,529
Trainable	—	15,102,529
Non-trainable	—	0

Note: _1 = “input1”, c2d = “convolutional2d”, mp2d = “ max_poolint2d”, c2d_1 = “convolutional2d1”, mp2d _1 = “max_poolint2d1”, c2d2 = “convolutional2d2 “, m2d_2 = “max_poolint2d2 “, *f*1 = “Flatten Layers”, *d*1 = “ dropout”, dt = “ dense1”, dns_1 = “dense2”, dot = “dropout1”. io1 = “3”, co1 = “ “, mpo2 = “ 32”, c2do1 = “64 “, mp2o1 = “64 “, c2o2 = “128 “, m2do = “ 128”,flo = “ 28800”, det5 = “512 “, dot5 = “512 “, dnst5 = “ 512”, *p*0 = “0”, *p*1 = “ 896”, *p*01 = “0”, *p*2 = “ 18496”, *p*02 = “0”, *p*3 = “ 73856”, *p*03 = “0”, *p*4 = “ 0”, *p*05 = “0”, d05 = “0”.

**Table 3:** Pretrained convolution neural network model (VGG-19).

Layer	Output	Parameter
input_2	[(*N*, 125, 125,3)]	0
b1-c1	(*N*, 125, 125, t1)	*P*1
b1-c2	(*N*, 125, 125, t1)	*P*1
b1-pool	(*N*, 62, 62, t1)	0
b2-c1	(*N*, 62, 62, t2)	*P*2
b2-c2	(*N*, 62, 62, t2)	*P*2
b2-pool	(*N*, 31, 31, t3)	0
b3-c1	(*N*, 31, 31, t4)	*P*3
b3-c2	(*N*, 31, 31, t4)	*P*3
b3-c3	(*N*, 31, 31, t4)	*P*3
b3_c4	(*N*, 31, 31, t4)	*P*3
b3-pool	(*N*, 15, 15, t4)	0
b4-c1	(*N*, 15, 15, t5)	*P*4
b4-c2	(*N*, 15, 15, t5)	*P*4
b4-c3	(*N*, 15, 15, t5)	*P*4
b4-c4	(*N*, 15, 15, t5)	*P*4
b4-pool	(*N*, 7, 7, t5)	0
b5-c1	(*N*, 7, 7, t5)	*P*5
b5-c2	(*N*, 7, 7, t5)	*P*5
b5-c3	(*N*, 7, 7, t5)	*P*5
b5-c4	(*N*, 7, 7, t5)	*P*5
b5-pool	(*N*, 3, 3, t5)	0
fla_1	(*N*, t5)	0
Dse-3	(*N*, dset5)	*P*5
Dt-2	(*N*, dttt5)	0
Dse-4	(*N*, dset5)	262656
Dt-3	(*N*, dt5)	0
Dse-5	(*N*, 1)	513
Total params:		22,647,361
Trainable params:		2,622,977
Nontrainable:		20,024,384

Note: b1-c1 and b1-c2 = “ block1_conv1 and block1_conv2”, b2-c1 and b2-c2 = “ block2_conv1 and block2_conv2”, b3-c1 and b3-c2 and b3-c3 and b3-c4 = ” block3_conv1 and block3_conv2 and block3_conv3 and block3_conv4”, b5-c1 and b5-c2 and b5-c3 and b5-c4 and b5-c5 = ” block5_conv1 and block5_conv2 and block5_conv3 and block5_conv4”. fla1 = ” flatten_1” *t*5 = 4608. dse3, dse4, dse5 = ” dense_3, dense_4, dense_5”, dt2 = ” droupout_2.

**Table 4:** Confusion matrix-based analyses.

Models	Accuracy	F1 score	Precision	Recall
Basic CNN	0.9397 ± 0.23	0.9397 ± 0.13	0.9397 ± 0.19	0.9397 ± 0.27
VGG-19 frozen	0.9486 ± 0.13	0.9482 ± 0.12	0.9456 ± 0.15	0.9480 ± 0.12
VGG-19 fine-tuned	0.9704 ± 0.06	0.9640 ± 0.06	0.9740 ± 0.07	0.9700 ± 0.03

**Table 5:** The performance report of the model classification.

	Precision	Recall	F1 score	Support
Healthy sample	0.97	0.96	0.96	4085
Malaria-sample	0.96	0.96	0.95	4173
Micro-average	0.97	0.97	0.97	8158
Macro-average	0.97	0.97	0.97	8158
Weighted-average	0.97	0.97	0.97	8158

## Data Availability

The data used to support the findings of this study are available from the corresponding author upon request.
